# Osteogenic cell fractions isolated from mouse tongue muscle

**DOI:** 10.3892/mmr.2015.3350

**Published:** 2015-02-13

**Authors:** KOJI HARADA, TOYOKO HARADA, TARANNUM FERDOUS, TAKANORI TAKENAWA, YOSHIYA UEYAMA

**Affiliations:** Department of Oral and Maxillofacial Surgery, Yamaguchi University Graduate School of Medicine, Ube, Yamaguchi 755-8505, Japan

**Keywords:** osteogenesis, stem cell, bone regeneration, tongue muscle, stem cell antigen-1

## Abstract

The use of stem cells represents a promising approach for the treatment of bone defects. However, successful treatments rely upon the availability of cells that are easily obtained and that appropriately differentiate into osteoblasts. The tongue potentially represents a source of autologous cells for such purposes. In the present study, the ability of stem cell antigen-1 (Sca-1) positive cells derived from tongue muscle to differentiate into osteoblasts was investigated. The tongue muscles were excised from Jcl-ICR mice and tongue muscle-derived Sca-1-positive cells (TDSCs) were isolated from the tongue muscle using a magnetic cell separation system with microbeads. TDSCs were cultured in plastic dishes or gelatin sponges of β-tricalcium phosphate (β-TCP) with bone differentiation-inducing medium. The expression of osteogenic markers (Runx2, osterix, alkaline phosphatase, fibronectin, osteocalcin, osteonectin and osteopontin) was investigated in cultured TDSCs by western blot analysis. The formation of mineralized matrices was examined using alizarin red S and Von Kossa staining. Bone formation was investigated in cultured TDSCs by hematoxylin-eosin staining and immunohistochemstry. In the present study, the expression of Sca-1 in mouse tongue muscle was demonstrated and TDSCs were isolated at high purity. TDSCs differentiated into cells of osteoblast lineage, as demonstrated by the upregulation of osteoblastic marker expression. The formation of mineralized matrices was confirmed by alizarin red S or Von Kossa staining *in vitro*. Bone formation was observed in the gelatin sponges of β-TCP, which were subsequently implanted under the skin of the backs of nude mice. These results suggested that TDSCs retain their osteogenic differentiation potential and therefore the tongue muscle may be used as a source of stem cells for bone regeneration.

## Introduction

Oral surgery frequently causes craniofacial bone defects in various situations, including trauma, infection, tumors, congenital malformations or degenerative skeletal diseases. To date, such bone defects have been repaired by the use of bone autografts and allografts (1,2); however, autografts and allografts require invasive surgery and the subsequent use of immunosuppressive agents. Therefore, the use of autologous osteogenic stem/progenitor cells may potentially overcome the disadvantages of autografts and allografts. Mesenchymal stem cells (MSCs) have been shown to be a potential cell source for bone-tissue engineering (3). Briefly, MSCs undergo osteogenic differentiation via a well-defined pathway following appropriate stimulation (4,5). However, the harvesting of bone marrow is an invasive procedure and therefore the burden on patients is great (1,6). Recently, it was reported that the tongue muscle may provide an additional source of autologous cells for cardiac regeneration. Briefly, Shibuya *et al* (7) isolated Sca-1-positive cells, which are considered stem cells, from tongue muscle and demonstrated that these positive cells were able to differentiate into beating cells similar to cardiomyocytes. Tongue muscle-derived Sca-1-positive cells (TDSCs), as well as MSCs, may have multipotent differentiation capacity and thus present a novel therapeutic tool with the potential to replace autologous tissue grafting for bone defects. However, to the best of our knowledge, few studies have utilized tongue muscle cells as a cell source for bone-tissue engineering. In the present study, TDSCs were isolated and their potential as a cell source for bone-tissue engineering was examined.

## Materials and methods

### Animals

Female Jcl-ICR mice (Japan SLC, Shizuoka, Japan) and female athymic nude mice with CAnN.Cg-Foxnlnu/CrlCrlj genetic backgrounds (CLEA Japan, Inc., Tokyo, Japan) were purchased at four weeks of age and bred in the Animal Center of Yamaguchi University (Ube, Japan). The animals were housed in plastic cages in a pathogen-free environment and kept in an air-conditioned room at 23±2°C with a relative humidity of 55±10% under a 12-h light/dark cycle. The mice were provided sterile water and food *ad libitum*. All experiments were approved by the Institutional Animal Care and Use Committee of Yamaguchi University. The study conformed to the Guide for the Care and Use of Laboratory Animals published by the US National Institutes of Health (NIH Publication no. 85-23, revised 1996; Bethesda, MA, USA).

### Immunohistochemistry

The 8-week-old mice were sacrificed through an overdose of Somnopentyl (200mg/kg; Merchk and Co., Inc., Whitehouse Station, NJ, USA), and the tongue of the mouse was resected using a surgical knife and was then fixed in 10% formalin neutral-buffer solution (Wako Pure Chemical Industries, Ltd., Osaka, Japan) and embedded in paraffin (Wako Pure Chemical Industries, Ltd., Osaka, Japan). Sections (4 *μ*m) were prepared from the paraffin blocks and mounted on slides. These sections were fixed and processed for immunostaining with anti-Sca-1 mouse monoclonal antibody (1:100; 130-092-529; BD Biosciences, Franklin Lakes, NJ, USA), anti-osteocalcin rabbit polyclonal antibody (1:100, sc-30044; Santa Cruz Biotechnology, Inc., Dallas, TX, USA), anti-SPARC (secreted protein acidic and rich in cysteine, also known as osteonectin) rabbit polyclonal antibody (1:100; sc-25574; Santa Cruz Biotechnology, Inc.), anti-osteopontin mouse monoclonal antibody (1:100; sc-21742; Santa Cruz Biotechnology, Inc.) and the appropriate peroxidase-conjugated goat anti-rabbit polyclonal or -mouse monoclonal immunoglobulin G (IgG) secondary antibody (1:100; sc-2005; Santa Cruz Biotechnology, Inc.). Negative controls were performed using non-specific IgG (1:100; sc-2072 or sc-2025; Santa Cruz Biotechnology, Inc.). The blocking and immunostaining were performed using the Dako Envision kit (Dako, Glostrup, Denmark) according to the manufacturer’s instructions. All specimens were counterstained with hematoxylin. The slides were subsequently examined under a bright-field microscope (BX51; Olympus Corp., Tokyo, Japan). A reddish-brown precipitate indicated a positive reaction.

### Isolation and expansion of TDSCs

TDSCs were obtained from the tongue muscle of 8-week-old female, Jcl-ICR mice. Briefly, mice were sacrificed and the tongue was removed, as described above. Enzyme solution containing 40 *μ*g/ml Liberase Blendzyme 3 (Roche Diagnostics GmbH, Mannheim, Germany) and 200 *μ*g/ml DNase I solution (Thermo Fisher Scientific, Waltham, MA, USA) in Dulbecco’s minimal essential medium (D-MEM; Sigma-Aldrich, St. Louis, MO, USA) was injected directly into the tongue with a 25-gauge needle (Terumo, Tokyo, Japan). Mouse tongues were incubated by agitation at 37°C for 1 h and dissociated with MACS Dissociator (Miltenyi Biotec, Bergisch Gladbach, Germany) completely. The dissociated tissue was centrifuged at 80.57 × g at 4°C for 2 min and the cell pellet was resuspended in phosphate-buffred saline without calcium or magnesium [PBS(-)]. The cell suspension was harvested and passed through a 100 *μ*m-mesh filter (Miltenyo Biotec). The cells were washed by adding MACS buffer [PBS(-) containing 0.5% bovine serum albumin and 2 mM EDTA; Miltenyi Biotec] and centrifuged at 80.57 × g at 4°C for 2 min. The supernatant was discarded and the cell pellet was resuspended in 50 ml MACS buffer. The cell suspension was passed through a 70 *μ*m-mesh filter (Miltenyi Biotec) and centrifuged at 1200 rpm at room temperature for 10 min. The supernatant was discarded, the cell pellet was resuspended in 10 ml MACS buffer and a cell suspension of 3.0×10^6^ nucleated cells in 80 *μ*l MACS buffer was prepared. FcR Blocking reagent (10 *μ*l; Miltenyi Biotec) was added and incubated at 4°C for 5 min. Subsequently, 10 *μ*l anti-Sca-1-fluorescein isothiocyanate (FITC) antibody was added and incubated at 4°C for 10 min. The cells were washed by the addition of 2 ml MACS buffer and centrifugation at 1200 rpm at 4°C for 10 min. The supernatant was discarded completely and the cell pellet was resuspended in 500 *μ*l MACS buffer. Sca-1 positive cells were separated from the cell suspension using a magnetic cell separation system with microbeads (autoMACS Pro Separator™; Miltenyi Biotec). Propidium iodide solution (final concentration, 1 *μ*g/ml) was added to the Sca-1 positive cells and the Sca-1 positivity of TDSCs was evaluated by flow cytometric analysis (FACSCalibur™; BD Biosciences). TDSCs were cultured in culture medium, which consisted of D-MEM supplemented with 5% fetal bovine serum (FBS; Thermo Fisher Scientific), 5% growth-stimulating medium (NH CFU-Medium^®^; Miltenyi Biotec), 100 U/ml penicillin, 100 *μ*g/ml streptomycin (Thermo Fisher Scientific) and 12 *μ*M l-glutamine (Invitrogen Life Technologies). Non-adherent cells were removed following 24 h of culture by washing with PBS and adding fresh culture medium. Every 3–4 days, cells were washed and fresh culture medium was added for a period of four weeks. Following four weeks of culture, cells were washed and trypsinized by incubation in 2 ml of 0.25% trypsin/1 mM EDTA (Thermo Fisher Scientific) for 2 min at 37°C. The trypsin/EDTA was neutralized by the addition of 10 ml culture medium and the cells (passage one) were replated in 10 ml culture medium in a 100-mm dish. Following one week of culture, cells were trypsinized and subcultured (passage two) at 1.0×10^5^ cells/100-mm dish in culture medium. The culture medium was replaced every three days. Following one further week, cells were trypsinized and either frozen at −80°C in TC-protecto cell freezing medium (DS Pharma Biomedical, Osaka, Japan) or expanded further by plating at 1.0×10^5^/100-mm dish in culture medium. Identical conditions were used for the subsequent passages.

### Cell growth analysis

To evaluate cell growth, clonal populations (derived from a single cell by limiting dilution) of TDSCs were plated at a density of 5×10^3^ cells/well and subcultured in a 96-well culture plate (BD Biosciences). Following two, four, six, eight, 10 and 12 days of culture, MTT was added to each well (25 *μ*l/well) and incubated for 4 h. The blue dye taken up by the cells was dissolved in dimethyl sulfoxide (100 *μ*l/well) and the absorbance was measured with a spectrophotometer (BioRad Laboratories, Hercules, CA, USA) at 490 nm. All assays were performed in triplicate.

### Osteogenic differentiation analysis

The osteogenic differentiation capacity of TDSCs was assessed by the measurement of alkaline phosphatase (ALP) activity, ALP staining, alizarin red S staining and Von Kossa staining under a bright-field microscope (BX51; Olympus Corp.). The cells were grown on six-well plates at a density of 5×10^5^ cells/well in bone differentiation-inducing medium (NH OsteoDiff Medium®; Miltenyi Biotec). The medium was replaced every two days.

### ALP activity

ALP activity was evaluated using fast *p*-nitrophenyl phosphate tablets (Sigma-Aldrich) according to the manufacturer’s instructions. Briefly, cells were seeded at a density of 1×10^4^ cells/well on six-well culture plates (BD Biosciences) in DMEM supplemented with 10% FBS. After 24 h, cells were treated with bone differentiation-inducing medium (Miltenyi Biotec). The treated cells were collected and lysed with 1X radioimmunoprecipitation assay buffer (Thermo Fisher Scientific). Subsequently, a Bradford protein assay sample (20 *μ*l) was prepared. The sample was reacted with buffered substrate (100 *μ*l) and the reaction was stopped by the addition of stop solution (0.2 M NaOH; 80 *μ*l). The relative quantity of reacted *p*-nitrophenyl was estimated from the absorbance at 405 nm (BioRad Laboratories) at days one, three, five, seven, 10, 14, 21 and 28 of culture. Each experiment was performed in triplicate.

### ALP staining

ALP staining was performed using a tartrate-resistant acid phosphatase and ALP double-stain kit (Takara Bio, Inc., Otsu, Japan) according to the manufacturer’s instructions. Briefly, cells were fixed with fixation solution (acetone/citrate buffer pH 5.4) for 5 min at room temperature and stained with a substrate for ALP (5-bromo-4-chloro-3-indolyl-phosphate/nitro blue tetrazolium; Sigma-Aldrich) for 45 min at room temperature. Cells were counterstained with methyl green for 5 min at room temperature.

### Alizarin red S staining for mineralized matrix

Cells were fixed with 70% ice-cold ethanol for 1 h at −20°C and stained with 40 mM alizarin red S solution (pH 4.2; Sigma-Aldrich) for 10 min at room temperature. Cells were dried following rinsing under running tap water. Red staining indicated mineral nodule formation.

### Von Kossa staining

Cells were fixed with absolute ethanol and stained using the Von Kossa method to detect mineral nodule formation *in vitro* using a Von Kossa Stain kit (Diagnostic BioSystems, Pleasanton, CA, USA) according to the manufacturer’s instructions. Cells were fixed with 70% ice-cold ethanol for 1 h at −20°C and stained with 5% silver nitrate for 60 min with exposure to ultraviolet light. Following washing with distilled water, cells were stained with 5% sodium thiosulfate for 3 min. Cells were subsequently rinsed under running tap water and stained with nuclear fast red stain for 5 min. Black staining was indicative of mineral nodule formation.

### Western blot analysis

Cells were lysed with radioimmunoprecipitation assay buffer and whole cell lysates were subjected to 10% SDS-PAGE and transferred onto polyvinylidene difluoride membranes (Thermo Fisher Scientific). The membranes were incubated with the anti-Sca-1 mouse monoclonal antibody (1:1,000), anti-c-kit rabbit polyclonal antibody (1:1,000; sc-168; Santa Cruz Biotechnology, Inc.), anti-osterix rabbit polyclonal antibody (1:1,000), anti-RUNX2 (runt-related transcription factor 2) rabbit polyclonal antibody (1:,000; sc-10758; Santa Cruz Biotechnology, Inc.), anti-fibronectin mouse monoclonal antibody (1:1,000; sc-59826; Santa Cruz Biotechnology, Inc.), anti-osteocalcin rabbit polyclonal antibody (1:1,000) and anti-osteopontin rabbit polyclonal antibody (1:1,000; sc-20788; Santa Cruz Biotechnology, Inc.). The membranes were then incubated with Novex^®^ alkaline-phosphatase-conjugated goat anti-rabbit polyclonal secondary antibody (WP20006; Thermo Fisher Scientific), or goat anti-mouse monoclonal secondary antibody (WP20007; Thermo Fisher Scientific) according to manufacturer’s instructions. The antibodies were detected using a chromogenic immunodetection system (WesternBreeze; Thermo Fisher Scientific) according to the manufacturer’s instructions. The anti-α-tubulin monoclonal antibody (Santa Cruz Biotechnology, Inc.) was used for the normalization of western blot analyses.

### Three-dimensional (3D) cell culture and histological evaluations

Cells were seeded into gelatin sponges of β-TCP (MedGel^®^ Scaffold; MedGel, Kyoto, Japan) by an agitated seeding method as it had been previously demonstrated that this method was effective for seeding cells homogeneously throughout porous 3D scaffolds (8,9). The cell-seeded gelatin sponges of β-TCP were cultured in tissue culture plates with bone differentiation-inducing medium at 37°C in a 5% CO_2_-95% air atmosphere for three weeks. Cell culture was performed for three weeks until 90% confluence was reached and the medium was replaced every three days. Subsequently, the cell-seeded gelatin sponges of β-TCP were transplanted subcutaneously into nude mice. In brief, a small incision was made using a knife into the dorsum of nude mice under general anesthetic (Sonnopentyl injection, 20 mg/kg). The cell-seeded gelatin sponges of β-TCP were inserted surgically beneath the skin and the incision sites were sutured using 3-0 silk (Alfresa Pharma Corporation, Osaka, Japan). All mice were monitored weekly. At 28 days post-transplantation, the cell-seeded gelatin sponges of β-TCP were resected with a surgical knife under general anesthesia (Somnopentyl, 20 mg/kg). The cell-seeded gelatin sponges of β-TCP were fixed in 10% neutral-buffered formalin solution, dehydrated, immersed in xylene and embedded in paraffin. The samples were cut into 4-*μ*m sections and stained with hematoxylin and eosin to histologically view on an optical microscope (BX51; Olympus Corp.).

## Results

### Sca-1-positive cells are located in the tongue muscle and may be isolated at high purity

Sca-1 expression was detected in the muscle of Jcl-ICR mouse tongues by immunohistochemical analysis. The majority of the expression of Sca-1 was localized to the tongue muscle rather than the tongue mucosa (Fig. 1). Cells were harvested from Jcl-ICR mouse tongue muscles and highly pure populations of Sca-1 positive cells were obtained using a magnetic cell separation system with microbeads. Briefly, 97.19% of cells in the Sca-1-positive fraction expressed Sca-1 (Fig. 2). TDSCs were able to be readily expanded in expansion medium and the doubling time was ~48 h. TDSCs exhibited a fusiform, fibroblast-like morphology (Fig. 3).

### Cultured Sca-1-positive cells differentiate into osteoblasts

The differentiation capacity of TDSCs was evaluated for osteoblast differentiation. TDSCs were cultured in bone differentiation-inducing medium supplemented with osteogenic induction components. TDSCs began to develop distinct mineralized nodules following 14 days in culture. The mineralized nodules were stained with alizarin red S or Von Kossa (Fig. 4). ALP activity was found to increase following treatment with bone differentiation medium until the activity peaked following 10 days of culture and subsequently decreased as determined by an assay with fast *p*-nitrophenyl phosphate tablets or cytochemical staining (Fig. 5).

Furthermore, western blot analysis of mesenchymal stem cell marker expression (Sca-1 and c-kit) and osteoblastic protein expression (osterix, Runx2, fibronectin, osteocalcin, osteonectin and osteopontin) was performed. As indicated in Fig. 6, TDSCs initially expressed mesenchymal stem cell markers and the expression of Sca-1 decreased following a peak at three days of culture. In addition, the expression of c-kit also decreased after peaking at the seventh day of culture. The expression of osteoblastic markers was increased by treatment with bone differentiation medium, although the majority began to decrease following a peak at 5–7 days of culture. Expression of osteocalcin was observed in 14–21 day-cultured cells.

### Sca-1-positive cells differentiate into bone in vivo

Subsequently, the *in vivo* differentiation potential of TDSCs was investigated. TDSCs were seeded into the gelatin sponges of β-TCP using an agitated seeding method and transplanted subcutaneously into nude mice. At 28 days post-transplantation, areas with bone-like morphology were observed in the gelatin sponges of β-TCP (Fig. 7A). Bone matrix expression was identified in the cells of these areas by immunohistochemical analysis. Cells in these areas produced osteocalcin, osteonectin and osteopontin (Fig. 7B–D).

## Discussion

In the present study, the potential of the tongue muscle as a cell source for bone-tissue engineering was evaluated, as stem cells, including satellite cells and muscle side population cells, exist in skeletal muscle tissue (10) and osterix overexpression enhances osteoblast differentiation of muscle satellite cells *in vitro* (11). Shibuya *et al* (7) previously succeeded at inducing cardiomyogenic differentiation of tongue muscle-derived stem cells. They used Sca-1 as a stem cell marker for isolating stem cells from mouse tongue muscle. Sca-1 was initially reported to be a cell surface marker of hematopoietic stem cells (12). However, several studies have since reported that multipotent stem cells derived from bone marrow (13) or skeletal muscle (14,15) also express Sca-1. Based on the results presented in the above reports, Sca-1 was selected as a stem cell marker for isolating stem cells from mouse tongue muscle in the present study. Notably, high expression levels of Sca-1 proteins were detected in the tongue muscles of Jcl-ICR mice. Following the method outlined by Shibuya *et al* (7), highly pure populations of Sca-1-positive cells were obtained from mouse tongue muscle using a magnetic cell separation system with microbeads.

It has been reported that osteoblasts synthesize the macromolecules of the bone matrix, including osteocalcin, osteonectin and osteopontin (16). Osteoblasts also express high levels of the membrane-bound enzyme ALP, which has a critical function in mediating matrix mineralization. Early in the process of cellular commitment to the osteoblastic phenotype ALP is expressed, whereas osteopontin and osteocalcin are expressed later during osteoblast differentiation (17–19). The treatment of TDSCs with bone differentiation-inducing medium resulted in the loss of stem cell markers c-kit and Sca-1. These TDSCs also began to express multiple osteogenic markers, including osterix, Runx2, fibronectin, osteocalcin, osteonectin and osteopontin, as well as the osteoblastic functions of mineralization and enhanced ALP activity. Furthermore, osteocalcin expression was found to be late in onset during osteoblast differentiation in the present study. These results demonstrated that the treatment of TDSCs with bone differentiation-inducing medium induced osteoblast differentiation *in vitro*.

TDSCs were able to form areas with bone-like morphology using the gelatin sponges of β-TCP as a scaffold. However, TDSCs were unable to form bone without the gelatin sponges of β-TCP (data not shown). Whether the gelatin sponges of β-TCP would be useful as a scaffold for bone formation remains to be elucidated. Therefore, the identification of a suitable scaffold for the formation of bone cells from TDSCs is required.

In conclusion, the present study provided evidence that TDSCs contained lineage-committed populations of pre-osteoblastic cells. TDSCs exhibited osteoblastic phenotypes in *in vitro* differentiation assays. Furthermore, TDSCs implanted subcutaneously into nude mice confirmed the results obtained from the *in vitro* differentiation assays, demonstrating that TDSCs were able to form areas with bone-like morphology in nude mice. However, prior to the clinical application of TDSCs, further experimental studies are required in order to elucidate the full benefits and side effects of this potential therapeutic approach.

## Figures and Tables

**Figure 1:** Sca-1 is expressed in the tongue muscle. (A and B) Hematoxylineosin staining, B is higher magnification of the box outlined in A. (C and D) Immunohistochemical staining with Sca-1 antibodies, D is higher magnification of the box outlined in C. The arrow indicates Sca-1-positive cells. Sca-1, stem cell antigen-1. Magnification: A and C, ×40; B and D, ×200.

**Figure 2:** Highly pure populations of Sca-1-positive cells isolated from mouse tongue muscle. Following magnetic cell sorting, 97.19% of cells in the Sca-1-positive fraction expressed Sca-1. PI negative indicated live cells and the reflecting pattern was used for the removal of dust and debris. Sca-1, stem cell antigen-1; PI, propidium iodide.

**Figure 3:** Growth curve of TDSCs identified by an MTT assay. The doubling time was ~48 h. TDSCs exhibited a fusiform, fibroblast-like morphology on day 2, as determined by phase-contrast microscopy (magnification, ×200). Values are expressed as the mean ± standard deviation, (n=6). TDSCs, tongue muscle-derived stem cell antigen-1 positive cells; OD, optical density.

**Figure 4:** *In vitro* osteoblast differentiation of TDSCs. TDSCs were induced to differentiate into osteoblasts for 28 days. Cells were stained with Von Kossa (left panels, black stain) or alizarin red S (right panels, red stain) for matrix mineralization (magnification, ×100). TDSCs, tongue muscle-derived stem cell antigen-1 positive cells.

**Figure 5:** *In vitro* ALP induction of tongue muscle-derived stem cell antigen-1 positive cells. ALP activity was increased following treatment of tongue muscle-derived Sca-1 positive cells with bone differentiation medium as determined by an ALP activity assay with fast *p*-nitrophenyl phosphate tablets or cytochemical staining. ALP, alkaline phosphatase.

**Figure 6:** TDSCs differentiate into bone following *in vitro* osteogenic induction. Western blot analysis revealed that TDSCs expressed mesenchymal stem cell markers (Sca-1 and c-kit) and their expression was decreased by the treatment with bone differentiation medium following a peak at three days of culture. Osteoblastic protein expression (osterix, Runx2, fibronectin, osteocalcin, osteonectin and osteopontin) was initially increased by treatment with bone differentiation medium, until expression levels peaked at 5–7 days of culture. Sca1, stem cell antigen-1; TDSCs, tongue muscle-derived Sca-1 positive cells.

**Figure 7:** TDSCs differentiate into bone *in vivo* following subcutaneous transplantation. (A) Hematoxylin and eosin staining indicated that TDSC implants exhibited bone-like morphology 28 days following transplantation. Immunohistochemistry of (B) osteocalcin, (C) osteonectin and (D) osteopontin (magnification, ×200). Arrows indicate positive staining (brown). TDSCs, tongue muscle-derived Sca-1 positive cells.
